The article "The Prevention of Senile Diabetes by Smart Wearable Health Monitoring Products" was retracted in 2023. Reasons: unreliable results or conclusions; lack of ethics approval or compliance; concerns about the data; concerns about the peer review.

# The Prevention of Senile Diabetes by Smart Wearable Health Monitoring Products

**DOI:** 10.1155/2022/5851199

**Published:** 2022-02-11

**Authors:** Wei Wei, Fangbo Li

**Affiliations:** Chinese Center for Health Education, Beijing, China

## Abstract

As a chronic disease, diabetes in the elderly patients is incurable and has a long treatment time, most of the symptoms are atypical, and onset is difficult to detect. This is among the challenging issues in front of doctors and paramedical stall and needed to be addressed on a priority basis as it poses a great threat to the health and life of the elderly. At present, the corresponding home medical products and emergency medical equipment cannot provide comprehensive and real-time services for monitoring physical conditions. At present, smart wearable health monitoring products are still in an emerging field. Relying on the advantages of internet technology, actively monitoring the physical condition of elderly diabetic patients is conducive to health protection. This article uses questionnaire surveys and experimental research methods to analyze the information source channels of the elderly diabetic patients interviewed for diabetes and their concerns about using smart wearable health monitoring products and compare their satisfaction with traditional blood glucose monitoring products and smart wearable health monitoring products. According to the investigation results of 50 elderly diabetes patients in P City,, they use TV, newspapers, and magazines to learn more about relevant information. They are mainly worried that they are unfamiliar with the product and will not use the process. Compared with traditional blood glucose monitoring products, smart wearable health monitoring products are satisfied, and degree is higher. Therefore, in order to better let elderly diabetic patients understand their physical condition, they can also effectively avoid the risk factors that may be suffered in life so that the disease can be effectively controlled. Various claims of the proposed scheme are verified through a rigorous evaluation process which is carried out in the form of numerous experiments. These results show that the proposed scheme is an effective way to resolve the aforementioned issue in the hospitals.

## 1. Introduction

In today's era, there is an aging population in many countries and regions, and this is an unavoidable trend. The increasing number of the elderly population also requires the entire medical system to pay much attention to the health problems of the elderly. Various chronic diseases, such as high blood pressure, hyperlipidemia, and diabetes, are common among the elderly. To a great extent, these diseases threaten the lives of the elderly. Among them, diabetes is a type of disease that is incurable, has a slow treatment time, and has a strong timeliness of treatment and medication. The current medical model in my country is quietly changing, from treatment-oriented to prevention-oriented, with self-monitoring. Therefore, health testing plays an important role in this aspect and provides certain guidance for other treatment methods. From the current point of view, more and more people are autonomously setting their sights on the emerging field of mobile health. Investigating its origin, mobile health is actually a mobile medical treatment and testing method, relying on the advantages of internet technology to provide patients with one-stop services and assistance in various aspects including examination, testing, evaluation, and treatment. In short, mobile health is the perfect combination of customized personalized medical services and mobile devices. Its outstanding advantages and characteristics are concentrated in the four major modules of information, service, application, and equipment. In some developed countries, mobile health started early and developed rapidly. For example, the United States and Japan have achieved the professional and refined process of mobile health, including mobile devices that can test ECG, blood sugar, and hearing. At present, high-tech intelligence is developing rapidly and has achieved fruitful results. Intelligent products are gradually applied in the field of medical and health care and the technological advantages of wearable devices are applied to the safety and health of the elderly so that they can benefit the elderly group and improve the quality of life of the elderly.

The article "The Prevention of Senile Diabetes by Smart Wearable Health Monitoring Products" was retracted in 2023. Reasons: unreliable results or conclusions; lack of ethics approval or compliance; concerns about the data; concerns about the peer review.

The related research results on health monitoring products and senile diabetes are very rich, but at present, it seems that the related research on the prevention of the onset of senile diabetes by smart wearable health monitoring products needs to be further improved. Zheng and others believed that the incidence of diabetes in the elderly is increasing and has become one of the three chronic diseases that endangers the health of Chinese residents [1]. Ni et al. proposed that monitoring blood sugar multiple times a day and regular health education are protective factors for hypoglycemia [2]. Wang proposed to rationally optimize the functions and user experience of wearable products and timely monitor the physical health and information feedback of the elderly [3]. Therefore, research on smart wearable health monitoring products for preventing the onset of senile diabetes still has great practical value.

At present, the corresponding home medical products and emergency medical equipment cannot provide comprehensive and real-time services for monitoring physical conditions. At present, smart wearable health monitoring products are still in an emerging field. Relying on the advantages of internet technology, actively monitoring the physical condition of elderly diabetic patients is conducive to health protection. This article uses questionnaire surveys and experimental research methods to analyze the information source channels of the elderly diabetic patients interviewed for diabetes and their concerns about using smart wearable health monitoring products and compare their satisfaction with traditional blood glucose monitoring products and smart wearable health monitoring products. Spend according to the survey results, they use TV, newspapers, and magazines to learn more about relevant information. They are mainly worried that they are unfamiliar with the product and will not use the process. Compared with traditional blood glucose monitoring products, smart wearable health monitoring products are satisfied, and degree is higher. Therefore, in order to better let elderly diabetic patients understand their physical condition, they can also effectively avoid the risk factors that may be suffered in life so that the disease can be effectively controlled. This article mainly includes the following aspects: introduces the status quo of elderly diabetic patients, related blood glucose monitoring products, wearable device products, and their problems and development advantages, research and analysis of the source channels of the interviewed elderly diabetic patients to understand the disease-related information, the use of concerns about smart wearable health monitoring products, comparative analysis of the satisfaction of traditional blood glucose monitoring products and smart wearable health monitoring products, and analysis of the corresponding results.

The article "The Prevention of Senile Diabetes by Smart Wearable Health Monitoring Products" was retracted in 2023. Reasons: unreliable results or conclusions; lack of ethics approval or compliance; concerns about the data; concerns about the peer review.

The rest of the paper is organized as follows. In Section 2, research on the prevention of senile diabetes by smart wearable health monitoring products is described along with real-world scenarios and practical examples. Moreover, current status of the elderly diabetic patients is reported to form the basis for the proposed model, whereas investigation and research on the prevention of senile diabetes by smart wearable health monitoring products are presented in Section 3 of the paper. In Section 4, the investigation and analysis of smart wearable health monitoring products on the prevention of senile diabetes are described followed by a comprehensive concluding remarks section.

## 2. Research on the Prevention of Senile Diabetes by Smart Wearable Health Monitoring Products

### 2.1. Current Status of Elderly Diabetic Patients

Most elderly people with diabetes have no obvious symptoms, are basically indistinguishable from ordinary people in appearance, and are easily overlooked and missed. Even many elderly patients miss the best period of treatment because they do not pay attention to check and monitor their physical condition, which leads to more serious consequences. Many elderly diabetic patients often first have related complications such as hypertension and cardiovascular disease, and in severe cases, they can also cause diseases with extremely high mortality such as cardiovascular and cerebrovascular diseases [4, 5].

At present, diabetes is a type of disease that is incurable, has a slow treatment time, and has a strong timeliness of treatment and medication. At present, the blood sugar control of diabetic patients is basically achieved by drugs and diet, which bring great inconvenience to elderly patients. In addition, due to the increase in age and the decline in self-control and memory, the elderly have increased the difficulty of treatment, so in their daily life, which aspects should be improved to improve the treatment effect of diabetes is particularly important [6, 7].

In the course of diabetes treatment, lifestyle habits are very important for blood sugar control. For elderly diabetic patients, diet, exercise, rest, and monitoring must be managed regularly, and the original bad habits must be managed and eradicated. Pay attention to the combination of work and rest. For elderly diabetic patients, healthy and fixed living habits are related to the development of their condition. However, due to the current diabetes medications and more attentional problems, most elderly patients cannot well control and restrain their own principles. Habits and, at the same time, due to the problems of blood glucose monitoring products and the fragmented presentation of blood glucose monitoring data, most elderly diabetic patients have aggravated the development of the disease due to untimely and unreasonable treatment [8, 9].

### 2.2. Related Blood Glucose Monitoring Products for Elderly Diabetic Patients

Diabetes is one of the most common chronic diseases in life, and many diabetic patients develop it unknowingly. Because of this, patients will use various products for diabetes treatment, assistance, and monitoring. An easy-to-use, simple, and user-friendly device can often help patients improve their health more effectively. With the continuous development of science and technology, smart products in the field of diabetes are constantly developing in a more convenient and humane direction. For example, there are corresponding medical management products on the market. Among them, blood glucose monitoring products can better monitor blood glucose levels and prevent the onset of senile diabetes in a timely and effective manner. Therefore, they have an important position in blood glucose control [10, 11].

The article "The Prevention of Senile Diabetes by Smart Wearable Health Monitoring Products" was retracted in 2023. Reasons: unreliable results or conclusions; lack of ethics approval or compliance; concerns about the data; concerns about the peer review.

The main products related to blood glucose monitoring on the market are blood glucose meters and blood glucose test strips. Among them, the traditional blood glucose monitoring equipment uses blood to detect the blood glucose content, which not only has certain risks in terms of hygiene but also the product experience is unsatisfactory. Blood glucose testing is also relatively easy to be affected by the external environment. Because the test results cannot truly reflect the true level of human blood glucose, some elderly diabetic patients cannot properly control their condition, leading to serious diabetic complications. Therefore, how to improve the effectiveness and ease of use of blood glucose testing products and how to design a more user-friendly, more portable, and smarter diabetes blood glucose monitoring equipment have become the main problems currently studied by many manufacturers [12, 13].

Sugar Nurse Smart Blood Glucose Monitor is a unique smart blood glucose meter in China, mainly targeting young people and the elderly. The whole product is composed of 4 parts: blood glucose meter, data display device (optional set), blood sampling pen, and sugar nurse application software. From the overall perspective of product design, portability and ease of operation are the main focus. Users can measure and record blood glucose meters through traditional blood sampling methods. The data will be synchronized to WeChat or app in real time and presented to users in the form of visual data. The advantages and disadvantages of this product are shown in Figure 1.

### 2.3. Smart Wearable Health Monitoring Products

#### 2.3.1. Overview of Smart Wearable Health Monitoring Products

At present, relevant research institutions in China have also carried out relevant research on telemedicine, electronic medical technology, and wearable health monitoring system. However, compared with developed countries, my country started late in the research and development of smart products for the elderly. There are few achievements in this field, and most of the experimental products have not yet been popularized. Smart wearable health monitoring products are currently one of the most promising products and will become a hot field in the future. At present, the wearable device on the market is still an emerging product, and its market, production scale expansion, and overall development and growth will require a certain amount of time and process. Of course, there are huge opportunities and challenges that follow. The elderly are more familiar with technology products that have entered daily life earlier, but at the same time, this group is very ignorant of emerging smart products. Although wearable devices have triggered a wave of companies entering the market, the industry is still in its infancy, and there are still many places worth exploring and discovering.

The article "The Prevention of Senile Diabetes by Smart Wearable Health Monitoring Products" was retracted in 2023. Reasons: unreliable results or conclusions; lack of ethics approval or compliance; concerns about the data; concerns about the peer review.

Health monitoring provides users with personalized, professional, and long-term care in their daily lives. It also conducts professional, continuous, and real-time monitoring of human health parameters, uses modern information methods to monitor and analyze indicators and evaluate analysis reports, provides suggestions and help, and enhances users' cognitive level and cognitive ability in self-monitoring and maintenance. It enables people to detect and control their physical health abnormalities, greatly reduces the harm caused by diseases and the economic burden caused by medical treatment, reduces family burden and social pressure, and greatly enhances people's living standards and quality.

Smart wearable health monitoring products monitor the physical condition of elderly patients in real time, generate corresponding specific information, and upload the data and detailed health analysis reports to the terminal device so that the patient can read the relevant information and understand their physical condition. The family members can also obtain the health information of the elderly at home in a timely manner. The hospital can also remotely use the data information on the terminal device to provide patients with appropriate treatment plans, daily precautions, and suggestions, which also reduces the distance between patients and the hospital. The system operation of smart wearable health monitoring products is roughly shown in Figure 2.

#### 2.3.2. Development Advantages of Smart Wearable Health Monitoring Products in the Medical and Health Field

The physical condition monitoring provided by wearable medical devices can slow down patients with chronic diseases to stay away from the ward and live a life similar to normal people, so they are the most stable customer group. Currently, wearable devices used for chronic disease monitoring have high user stickiness. The main user groups of these products are people with diabetes and cardiovascular diseases.

Therefore, smart wearable health monitoring products have certain development advantages in the medical and health field. One is to have a relatively stable customer base. At present, the main user groups of smart wearable health monitoring products are people with diabetes and cardiovascular diseases. The characteristics of these diseases are incomplete cure, high treatment costs, and long-term monitoring and management. The second is that, in our country, the aging of the population has led to increasing medical demand in the society, so the development of mobile medical care is the general trend. The third is the rapid advancement of the Internet of Things and big data technology to provide strong technical support for mobile medical care. The fourth is that the Chinese government has issued a number of related policies and documents to clearly support and encourage the development of mobile medicine [14, 15].

The article "The Prevention of Senile Diabetes by Smart Wearable Health Monitoring Products" was retracted in 2023. Reasons: unreliable results or conclusions; lack of ethics approval or compliance; concerns about the data; concerns about the peer review.

### 2.4. Optimal Configuration of Health Monitoring Sensors

In order to optimize the configuration of health monitoring sensors, first, understand the modal motion energy. While the target modal linearity is obtained, the modal energy of the measuring point structure is larger. The formula of the residual coefficient of the effective independent driving point that defines the modal motion energy of the element stiffness is as follows:

(1) $$\begin{array}{c} D_{DPR}=\sum_{h=1}^{k}\frac{\phi_{uh}^{2}}{\theta_{uh}^{2}}. \end{array}$$

After weighting *D*_*DPR*_, the formula for the effective independent allocation matrix is as follows:

(2) $$\begin{array}{c} F_{a}=\phi_{r}{\left[\phi_{r}^{Y}\phi_{r}\right]}^{-1}\phi_{r}^{Y}D_{DP\;R}. \end{array}$$

Among them, *ϕ*_*uh*_ is the *h*th target modal vibration shape of the *u*th unit; *θ*_*uh*_ is the *h*th target modal frequency of the *u*th unit.

## 3. Investigation and Research on the Prevention of Senile Diabetes by Smart Wearable Health Monitoring Products

### 3.1. Questionnaire Design Process

The subjects of the questionnaire survey were 50 elderly diabetic patients in P city. Through interviews or the issuance of paper questionnaires, recovery, and quantitative analysis of the information filled in by users, the conclusion of the questionnaire is reached.

1. The preliminary preparation of the questionnaire considers that the number of questions should be as simple as possible to avoid fatigue or incomprehension of the interviewees.
2. The questionnaire is distributed through on-site questionnaires to fill in the questionnaires. A total of 50 questionnaires are distributed (100 villagers), and 50 valid questionnaires are returned. The questionnaire recovery rate is 100%.
3. Questionnaire analysis: the collected questionnaire information is sorted out, and the required information data are obtained. The results of the questionnaire were analyzed. The results of the analysis included the information source channels of the elderly diabetic patients interviewed, their concerns about the use of smart wearable health monitoring products, and their satisfaction with traditional blood glucose monitoring products and smart wearable health monitoring products. Some of the results of the questionnaire are as follows.

The article "The Prevention of Senile Diabetes by Smart Wearable Health Monitoring Products" was retracted in 2023. Reasons: unreliable results or conclusions; lack of ethics approval or compliance; concerns about the data; concerns about the peer review.

### 3.2. Questionnaire Survey Content

- The first part is a survey of 50 interviewed elderly diabetic patients on the sources of diabetes information
- The second part is a survey of 50 respondents' concerns about using smart wearable health monitoring products
- The third part is to compare the satisfaction of traditional blood glucose monitoring products and smart wearable health monitoring products
- The fourth part is to sort out the information collected in the questionnaire, learn about the respondents' understanding of land resource protection policies and related laws, and compare their satisfaction with traditional blood glucose monitoring products and smart wearable health monitoring products

## 4. The Investigation and Analysis of Smart Wearable Health Monitoring Products on the Prevention of Senile Diabetes

Focusing on smart wearable health monitoring products, a questionnaire survey of 50 elderly diabetic patients was conducted, and the analysis results were finally obtained.

### 4.1. Analysis of the Information Source Channels of the Elderly Diabetic Patients Interviewed for Diabetes

First, understand the sources of daily information about diabetes for these 50 elderly diabetic patients, and make an analysis, as shown in Table 1 and Figure 3.

It can be seen from Figure 3 that, in the information channels for the interviewed elderly diabetic patients to understand diabetes, TV and newspapers and magazines accounted for a larger proportion, respectively, 0.36 and 0.25. Therefore, they understand that daily information about diabetes mainly comes from newspapers, magazines, and television.

### 4.2. Analysis of Concerns about the Use of Smart Wearable Health Monitoring Products among Interviewed Elderly Diabetic Patients

After the interview, I learned about the concerns of the interviewed elderly diabetic patients about using smart wearable health monitoring products and made an analysis, as shown in Table 2 and Figure 4.

It can be seen from Figure 4 that, among the concerns of the interviewed elderly diabetic patients about the use of smart wearable health monitoring products, the proportions of being unfamiliar with the product and not knowing the use process are relatively large, respectively, 0.29 and 0.34. Therefore, the interviewed elderly diabetic patients are mainly worried about the use of smart wearable health monitoring products that they are unfamiliar with the product and unclear about the use process.

The article "The Prevention of Senile Diabetes by Smart Wearable Health Monitoring Products" was retracted in 2023. Reasons: unreliable results or conclusions; lack of ethics approval or compliance; concerns about the data; concerns about the peer review.

### 4.3. Comparative Survey Analysis of Respondents' Satisfaction with Traditional Blood Glucose Monitoring Products and Smart Wearable Health Monitoring Products

After the interview, understand the respondents' satisfaction with traditional blood glucose monitoring products and smart wearable health monitoring products, and make a comparative analysis, as shown in Table 3 and Figure 5.

It can be seen from Figure 5 that, after showing the use process of smart wearable health monitoring products, a total of 21 respondents were very satisfied and satisfied with using traditional blood glucose monitoring products. As for smart wearable health monitoring products, there were 33 people. Therefore, respondents are more satisfied with smart wearable health monitoring products than using traditional blood glucose monitoring products.

## 5. Conclusion and Future Directives

Under the current social background, the aging population and the rapid increase of patients with chronic diseases have brought severe tests and huge challenges to all aspects of today's society. At the same time, with the continuous development of science and technology, more and more smart products are used in the field of health care, providing real-time health monitoring services for patients with various chronic diseases, rather than relying on hospitals and certain medical institutions. It provides more effective ways to monitor the health of the elderly. The data results generated under the support of big data technology can effectively help doctors accurately assess the disease, find abnormal changes in the disease, adjust the diagnosis and treatment plan, and really help the treatment of the disease. Therefore, it is necessary to do a good job of propaganda work to provide adequate guidance and assistance to elderly diabetic patients so that elderly friends can do self-monitoring and self-prevention at home, so as to provide more convenience to their daily lives. Therefore, the research on the prevention of the onset of senile diabetes by smart wearable health monitoring products is very valuable in both the medical field and the science and technology field, and it has a broad space for development and bright prospects. This article uses questionnaire surveys and experimental research methods to analyze the information source channels of the elderly diabetic patients interviewed for diabetes and their concerns about using smart wearable health monitoring products and compare their satisfaction with traditional blood glucose monitoring products and smart wearable health monitoring products. Spend according to the survey results, they use TV, newspapers, and magazines to learn more about relevant information. They are mainly worried that they are unfamiliar with the product and will not use the process. Compared with traditional blood glucose monitoring products, smart wearable health monitoring products are satisfied, and degree is higher.

The article "The Prevention of Senile Diabetes by Smart Wearable Health Monitoring Products" was retracted in 2023. Reasons: unreliable results or conclusions; lack of ethics approval or compliance; concerns about the data; concerns about the peer review.

This work can be extended further by implementing it in the real environment of hospitals. Additionally, size of the wearable devices can be further minimized to improve the confidence level of various patients in wearing these devices 24 hours a day.

## Figures and Tables

**Figure 1:** Advantages and disadvantages of this product.

**Figure 2:** The system operation of smart wearable health monitoring products.

**Figure 3:** Analysis of the sources of information on diabetes by interviewed elderly diabetic patients.

**Figure 4:** Analysis of the concerns of interviewed elderly diabetic patients about using smart wearable health monitoring products.

**Figure 5:** Comparative survey and analysis of respondents' satisfaction on the traditional blood glucose monitoring products and smart wearable health monitoring products.

**Table 1:** Analysis of the sources of information on diabetes by interviewed elderly diabetic patients.

Channel	Data
Television	0.36
Newspapers and magazines	0.25
Radio	0.17
Hospital	0.13
Family and friends	0.11

**Table 2:** Analysis of the concerns of interviewed elderly diabetic patients about using smart wearable health monitoring products.

Concern	Data
Cost	0.16
Privacy security	0.18
Lack of understanding	0.29
Do not know how to use	0.34
Else	0.03

**Table 3:** Comparative survey and analysis of respondents' satisfaction on the traditional blood glucose monitoring products and smart wearable health monitoring products.

Project	Traditional blood glucose monitoring products	Smart wearable health monitoring products
Very satisfied	9	15
Satisfied	13	18
General	20	10
Dissatisfied	8	7

## Data Availability

The data underlying the results presented in this study are available within the manuscript.
